The article "Post-mastectomy benign lymphangioendothelioma of the skin following chronic lymphedema for breast carcinoma: a teaching case mimicking low-grade angiosarcoma and masquerading as Stewart-Treves syndrome" was published in 2014. Journal: Diagn Pathol.

# Post-mastectomy benign lymphangioendothelioma of the skin following chronic lymphedema for breast carcinoma: a teaching case mimicking low-grade angiosarcoma and masquerading as Stewart-Treves syndrome

**DOI:** 10.1186/s13000-014-0197-5

**Published:** 2014-10-29

**Authors:** Sohsuke Yamada, Yoko Yamada, Miwa Kobayashi, Ryosuke Hino, Aya Nawata, Hirotsugu Noguchi, Motonobu Nakamura, Toshiyuki Nakayama

**Affiliations:** Departments of Pathology and Cell Biology, School of Medicine, University of Occupational and Environmental Health, 1-1 Iseigaoka, Yahatanishi-ku, Kitakyushu, 807-8555 Japan; Departments of Dermatology and Immunology, School of Medicine, University of Occupational and Environmental Health, Kitakyushu, Japan

**Keywords:** Benign lymphangioendothelioma (BL), Skin, Angiosarcoma, Chronic lymphedema, Stewart-Treves syndrome, MIB-1

## Abstract

Benign lymphangioendothelioma (BL) represents a very rare lymphatic vascular proliferation. Our aim is to be aware that owing to its characteristic features, pathologists can easily misinterpret it as cutaneous low-grade angiosarcoma when examining only small specimens. In the present case, multiple small and yellowish to reddish soft nodules were noticed in the edematous left arm of a 54-year-old Japanese female 4 years after the radical mastectomy with axillary lymph nodes dissection and following radiotherapy to the chest for the left breast carcinoma. The biopsy specimen showed an ill-defined lesion composed of a proliferation of irregular and sometimes anastomosing vascular structures in the dermis, lined by endothelial cells having mildly hyperchromatic and pleomorphic nuclei, but no mitotic figures. As the lesion grew within deeper dermis, these proliferating vessels dissected dermal collagenous bands, occasionally arranged in low-papillary projections and/or characteristic hobnail cytomorphology. We first interpreted it as low-grade angiosarcoma following chronic lymphedema due to the operation, i.e., the so-called Stewart-Treves syndrome. Although additional treatments were performed for 7 years, she had neither local invasion nor metastases of these tumors, respectively, and was alive and well. Retrospective immunohistochemical findings demonstrated that these mildly atypical endothelial cells were strongly positive for lymphatic vessel endothelial hyaluronan receptor (LYVE)-1 as well, and MIB-1 labeling index was less than 1%. Therefore, we finally made a diagnosis of BL of the skin. MIB-1 labeling index might be useful and adjunctive aids for reaching the correct diagnosis of cutaneous BL, especially in case of small or inadequate specimens.

**Virtual Slides:** The virtual slide(s) for this article can be found here: http://www.diagnosticpathology.diagnomx.eu/vs/13000_2014_197

The article "Post-mastectomy benign lymphangioendothelioma of the skin following chronic lymphedema for breast carcinoma: a teaching case mimicking low-grade angiosarcoma and masquerading as Stewart-Treves syndrome" was published in 2014. Journal: Diagn Pathol.

## Background

Among all sarcomas, angiosarcomas are rare, accounting for merely less than 1% [1]. Enzinger and Weiss have classified them as follows: (a) cutaneous angiosarcoma associated with lymphedema; (b) cutaneous angiosarcoma unassociated with lymphedema; (c) angiosarcoma of the breast; and (d) angiosarcoma of deep soft tissue [1]. Intriguingly, about 90% of all (a) angioosarcomas associated with chronic lymphedema occur after mastectomy for breast cancer [1,2]. Actually, Stewart and Treves first reported the development of angiosarcoma arising on longstanding lymphedematous extremities, due to axillary lymph nodes dissection following a radical mastectomy, named as the so-called Stewart-Treves syndrome, in 1948 [3]. Clinically, this disease is characterized by red to blue and firm nodules and/or plaques on the affected extremities [2,3]. To date, more than 400 cases of Stewart-Treves syndrome have been described in the literature, and the patients have a very poor prognosis, complicated with recurrence, distant metastases, and very early death within 2 years [3,4]. It is also noteworthy that the prevalence is estimated at about 0.45% in patients with Stewart-Treves syndrome who survive longer than post-operative 5 years [4], and in fact, that very few long-term survivors have been recognized [1,2].

By contrast, among the lymphatic neoplasms, benign lymphangioendothelioma (BL) represents a very rare lymphatic vascular proliferation, histopathologically mimicking other malignant vascular neoplasms, such as cutaneous low-grade angiosarcoma, and readily misdiagnosed as it [5]. BL, also named as acquired progressive lymphangioma, was first described by Wilson Jones *et al.* in 1990 [6,7], and only 40 cases have been reported in the English-language literature [7,8]. Clinically, a typical lesion is a solitary and well-circumscribed red or bruise-like macule, plaque or nodule, which can be variably located on the breast, arm, face, scalp, or thigh [5-8]. BL has a tendency to present in middle-aged to elderly adults and particularly evolve slowly over years [5,7,8]. Moreover, the BL lesions are usually asymptomatic but occasionally have a predisposing factor, e.g., radiotherapy, trauma, arteriography, or tick bite [8]. One of the most important differential diagnosis is with low-grade angiosarcoma, since BL shares with angiosarcoma the histopathological presence of extensive dissection of collagen bundles [5,8]. Thus, it is critical to establish an accurate initial diagnosis whether benign or malignant by biopsy specimens, however, previous studies have indicated the somewhat difficulties of correct characterization of BL [8,9].

The article "Post-mastectomy benign lymphangioendothelioma of the skin following chronic lymphedema for breast carcinoma: a teaching case mimicking low-grade angiosarcoma and masquerading as Stewart-Treves syndrome" was published in 2014. Journal: Diagn Pathol.

We report an extremely rare case of post-mastectomy cutaneous BL following chronic lymphedema, easily confused with low-grade angiosarcoma, so-called Stewart-Treves syndrome.

## Materials and methods

The patient was a 45-year-old Japanese woman. The time interval from the first and follow-up biopsy was 7 years. The tumor biopsy specimens after fixation in 10% neutral buffered formalin were embedded in paraffin for histological or immunohistochemical examinations. We counted the number of proliferating lymphatic vessels in 10 randomly selected fields of not only tumor but non-tumor areas per section (original magnification: ×400) [10,11]. All immunohistochemical stainings were carried out using Dako Envision kit (Dako Cytomation Co., Glostrup, Denmark) according to the manufacturer’s instructions. 1]. Furthermore, the distribution of the staining with MIB-1 (Ki67; DAKO) in the tumor was assessed semi-quantitatively, counted at high power (original magnification: ×400) magnification. At least 1,000 nuclei were counted in each section. The MIB-1 labeling index was presented as number of positive nuclei per 1,000 nuclei counted [12].

All histological and immunohistochemical slides were evaluated by two independent observers (certified surgical pathologists in our department) [10-12]. Agreement between observers was excellent (>0.9) for all antibodies investigated as measured by interclass correlation coefficient. For the few instances of disagreements, a consensus score was determined by the third board-certified pathologists in our department [10-12].

All values are expressed as the means ± SE. Significant differences were analyzed using Student’s *t*-test. Values of *P* <0.05 were considered to be statistically significant.

## Case presentation

### Clinical summary

The patient had a history of left breast carcinoma, diagnosed as invasive ductal carcinoma but unknown detailed histological features, 4 years ago. She underwent a radical mastectomy with axillary lymph nodes dissection and following radiotherapy to the chest for it. There was no history of immunosuppressive disorders, use of immunosuppressive medications, or unusual infections, including acquired immunodeficiency syndrome (AIDS).

She suffered from chronic lymphedema of the left arm supervened shortly after the operation (Figure 1A) and noticed multiple small and yellowish to reddish soft nodules, measuring up to 6 mm in the edematous left arm (Figure 1B). Since the number of those lesions was gradually increasing, a biopsy was performed. Moreover, interleukin-2 immunotherapy, additional radiotherapy (to the chest) and adjuvant chemotherapy using low-dose docetaxel were done for post-operative 7 years, under the initial diagnosis of low-grade angiosarcoma following longstanding lymphedema due to the radical mastectomy with axillary lymph nodes dissection for the breast carcinoma, i.e., the so-called Stewart-Treves syndrome, based on the initial clinicopathological features. Laboratory data, including blood cell count and chemistry, were within normal limits, except for modestly high level of hemoglobin A1c (HbA1c; 6.1 mg/dL), and there was no evidence of tumor or tumor-like lesions in the CT scannings of chest and abdomen. Anti-human immunodeficiency virus (HIV) antibodies were completely negative. Within the post-operative 7 years with additional treatment of interleukin-2 immunotherapy and chemo-radiotherapy, partial remission and neogenesis of the above small nodules were repeatedly seen. Very surprisingly, the patient had neither local invasion nor metastases of these lesions, respectively, and was alive and well at 5 years after the final chemotherapy. Furthermore, other skin lesions including those at the mastectomy site have never appeared.

The article "Post-mastectomy benign lymphangioendothelioma of the skin following chronic lymphedema for breast carcinoma: a teaching case mimicking low-grade angiosarcoma and masquerading as Stewart-Treves syndrome" was published in 2014. Journal: Diagn Pathol.

**Figure 1:** **Clinical finding of this BL. (A, B)** The patient suffered from chronic lymph edema of the affected left arm supervened shortly after the radical mastectomy with axillary lymph nodes dissection **(A)** and noticed multiple small and yellowish to reddish soft nodules (**A**, arrows), measuring up to 6 mm in the edematous left arm **(B)**. The number of those lesions was gradually increasing up. Bar = 10 mm.

### Pathological findings

The first small biopsy specimen (Figure 2A) showed an ill-defined lesion predominantly composed of a significant proliferation of irregular and sometimes anastomosing vascular structures containing no red blood cells mostly in the middle to lower layer of dermis (tumor: 24.5 ± 2.9 per 1 high power fields vs. non-tumor: 2.7 ± 0.4 per 1 high power fields; *P* <0.0001) (Figure 2A). Few lesions involve the superficial dermis, and extension into the subcutaneous fat was absent (Figure 2A). These vascular channels were lined by modestly atypical endothelial cells having mildly hyperchromatic and pleomorphic nuclei, but no apparent mitotic figures (Figure 2B). As the lesion grew within deeper dermis, these proliferating vascular channels dissected dermal collagenous bundles, occasionally arranged in low-papillary projections and/or characteristic hobnail or multi-layered cytomorphology (Figure 2B). Surrounding lymphocytic infiltrate was not evident. On the other hand, the covering epidermis exhibited mild acanthosis and modestly elongated thickened rete ridge without any evidence of atypical changes (Figure 2A). Based on these features, we first diagnosed it as low-grade angiosarcoma following chronic lymphedema due to the radical mastectomy, i.e., the so-called Stewart-Treves syndrome. However, the follow-up biopsy specimens from the affected left arm demonstrated no evidence of any remarkable changes on histopathological findings, very similar to those of the above first biopsy sample. Immunohistochemically, these proliferating endothelial cells were positive for CD31 (DAKO, diluted 1:20) (Figure 3A), factor VIII-related antigen (DAKO, diluted 1:30), CD34 (IMMUNOTECH, Marseille, France, diluted 1:50), and Podoplanin (D2-40; Nichirei Bioscience Co., Tokyo, Japan, diluted 1:1) on the first biopsy specimen. Furthermore, the tumor cells of both the first and follow-up biopsy specimens showed strong immunohistochemical expression of lymphatic vessel endothelial hyaluronan receptor (LYVE)-1 (LYVE-1; R&D Systems, Inc., Minneapolis, MN, USA, diluted 1:320) (Figure 3A) and lower MIB-1 (Ki67; DAKO, diluted 1:50) labeling index, less than 1% (0.3%) (Figure 3B). There was no immunohistochemical expression of human herpes virus (HHV)-8 (HHV-8; Santa Cruz Biotechnology, Santa Cruz, CA, USA, diluted 1:100). Therefore, we confirmed that these mildly proliferating endothelial cells were derived from lymphatic vessels, and finally made a diagnosis of post-mastectomy BL of the skin following chronic lymphedema, based on the clinicopathological findings including its unusually benign clinical course.

The article "Post-mastectomy benign lymphangioendothelioma of the skin following chronic lymphedema for breast carcinoma: a teaching case mimicking low-grade angiosarcoma and masquerading as Stewart-Treves syndrome" was published in 2014. Journal: Diagn Pathol.

**Figure 2:** **Microscopic examination of the first biopsy specimen. (A)** The first small biopsy specimen (H&E stains, inset) revealed an ill-defined lesion predominantly composed of a proliferation of irregular and sometimes anastomosing vascular structures containing no red blood cells mostly in the middle to lower layer of edematous dermis. Few lesions involve the superficial dermis, and extension into the subcutaneous fat was absent (inset). The covering epidermis exhibited mild acanthosis and modestly elongated thickened rete ridge without any evidence of atypical changes (H&E stains). Bars =1 mm. **(B)** On high-power view (H & E stains), these vascular channels were lined by modestly atypical endothelial cells having mildly hyperchromatic and pleomorphic nuclei, but no apparent mitotic figures. As the lesion grew within deeper dermis, these proliferating vascular channels dissected dermal collagenous bundles, occasionally arranged in low-papillary projections (inset) and/or characteristic hobnail or multi-layered cytomorphology (inset). Surrounding lymphocytic infiltrate was not evident. Bar = 200 μm.

**Figure 3:** **Immunohistochemical examination of the first biopsy specimen. (A)** These modestly atypical endothelial cells were positive for CD31, but strongly positive for LYVE-1. **(B)** The tumor cells showed a much lower MIB-1 labeling index, less than 1%. Bars =50 μm.

The article "Post-mastectomy benign lymphangioendothelioma of the skin following chronic lymphedema for breast carcinoma: a teaching case mimicking low-grade angiosarcoma and masquerading as Stewart-Treves syndrome" was published in 2014. Journal: Diagn Pathol.

## Discussion

The most important differential diagnosis in the present BL case is with a low-grade angiosarcoma following post-mastectomy chronic lymphedema, i.e., the so-called Stewart-Treves syndrome. Clinically, the average time between radical mastectomy and angiosarcoma progression is reported to 12.5 years, displaying various features, such as red-blue firm nodules, plaques, blood blisters or ulcer formation, usually in the background of more than 10-years lymphedema [1,2], unlike the present case. In addition, extremely rare long-term survivors with Stewart-Treves syndrome are reported to have early amputation of the affected extremity [2]. Our case actually showed neither local invasion nor metastases within the post-operative 7 years with additional treatment of immunotherapy and adjuvant chemo-radiotherapy, but was also alive and well at 5 years after the final chemotherapy, manifesting as overtly benign clinical behavior. In contrast, BL occurring in a patient with chronic lymphedema after mastectomy is much rarer than Stewart-Treves syndrome. Indeed, although an extraordinary case of BL in a 48-year old woman is reported, appearing in the breast skin close to a mastectomy scar 3 years after surgery for invasive ductal carcinoma, the authors have never referred to chronic lymphedema [13]. Since it remains unclear whether the chronic lymedema is a predisposing factor for the BL lesions [8], further studies are thus needed to address the disease developing mechanism after collecting and investigating a much larger number of BL cases clinicopathologically examined. In fact, more recently, there have been some evidences about that BL is not a true neoplasm but rather a lymphatic vascular malformation by reason of the absence of Wilms tumor 1 (WT-1) expression [14]. BL occasionally presents as multiple nodular and/or papular lesions, as in the current case not only synchronous but metachronous [5,13]. In this context, we for the first time report an extremely rare case of post-mastectomy cutaneous BL following chronic lymphedema in the affected arm, easily confused with low-grade angiosarcoma, so-called the Stewart-Treves syndrome.

As to the present case, the pathologists first made a diagnosis as suspicious or suggestive of low-grade angiosarcoma. As shown in Figure 2, BL is characterized by the presence of irregular, tortuous and anastomosing endothelial-lined vessels, showing hobnail cytomorphology, and dissecting between dermal collagen bundles as the lesion permeates the deep dermis, similar to invasive features of malignant neoplasms. Moreover, it is possible that a small amount of the biopsy specimen further results in the misdiagnosis of a malignant angiosarcoma-like lesion. A tentative diagnosis of vascular tumor with malignant potential should be borne in mind at the very least, whenever pathologists encounter dermal collection of vascular vessels with an invasive growth pattern. However, in addition to the suspicion of no clinical malignancy, a detailed histopathological study can retrospectively reveal that the vascular channels usually devoid of red blood cells display neither cellular nor poorly differentiated areas, and that the lining endothelial cells have mild cellular atypia with absence of prominent nuclear pleomorphism or mitotic figures [5-9,13], as presented here. By contrast, we propose that the MIB-1 labeling index should be a useful and adjunctive aid for BL to distinguish from low-grade angiosarcoma, as well as the number of mitoses or highly atypical cells. Even a small amount of the biopsy specimen demonstrated a very low (less than 1%) MIB-1 positivity (Figure 3B), corresponding to the few previous immunohistochemical studies of BLs [13]. Further investigation with more clinicopathological samples of cutaneous BL, is necessary to confirm the importance of this well-known proliferative indicator. Nevertheless, since the primary biopsy sampling in the current case was adequate, BL of the skin might not be problematic for one of the initial differential diagnoses. Furthermore, the above clinically good course plus pathologically modestly atypical tumor cells seem to provide enough information for pathologists to recommend careful follow-up but not additional treatments.

The article "Post-mastectomy benign lymphangioendothelioma of the skin following chronic lymphedema for breast carcinoma: a teaching case mimicking low-grade angiosarcoma and masquerading as Stewart-Treves syndrome" was published in 2014. Journal: Diagn Pathol.

Among malignant to benign tumors, histopathologically differential diagnoses include vascular vessel proliferations in the dermis, such as patch-stage Kaposi’s sarcoma, retiform hemangioendothelioma, lymphangioma circumscriptum, or lymphangiomatous papules of the skin, respectively [2,5-9,13]. Immunohistochemical analyses partly resolve the distinction from the first Kaposi’s sarcoma easily, since Kaposi’s sarcoma is often identified in HIV-infected patients and is usually positive for HHV-8 [14], unlike in the present case. Furthermore, strong immunohistochemical expression of antibody against novel lymphatic marker, LYVE-1 (Figure 3A), might allow discrimination of BL from malignant vascular tumors [15], although it will be intriguing to see whether LYVE-1 immunoexpression pattern have reliable roles in this regard. However, it is also important to histologically recognize concomitant lymphoplasmacytic or lymphocytic infiltration of the dermal interstitium in Kaposi’s sarcoma or retiform hemangioendothlioma, in contrast to BL [1,9]. As to the benign lymphatic vessels proliferation, including lymphangioma circumscriptum or lymphangiomatous papules, the features of hobnail morphology and/or anastomosing or papillary structures are never as specific or pronounced as those observed in BL [5-9,13,14]. In fact, lymphangioma is predominantly composed of numerous dilated but not irregular-shaped lympatic vessels [5-9,13].

## Conclusion

We reported an extremely rare case of post-mastectomy BL of the skin following chronic lymphedema, histopathologically mimicking low-grade angiosarcoma and masquerading as the so-called Stewart-Treves syndrome. The present case was tentatively misdiagnosed as malignancy on the examination of the first biopsy specimen, since its section showed an ill-defined lesion composed of a proliferation of irregular and sometimes anastomosing vascular structures lined by mildly atypical endothelial cells. Additionally, these proliferating vessels dissected dermal collagenous bundles in the middle to lower layer of dermis, as the lesion grew within deeper dermis, arranged in low-papillary projections and/or characteristic hobnail cytomorphology. All pathologists should be aware that its characteristic features could easily lead to a misdiagnosis of low-grade angiosarcoma. Furthermore, we suggest that MIB-1 labeling index might be useful and adjunctive aids for recognizing no evidence of malignancy and reaching the correct diagnosis of cutaneous BL, as well as modestly atypical lining endothelial cells with mildly pleomorphic nuclei, but no apparent mitotic figure, especially in case of small or inadequate specimens. In this context, the present case report should interest the scientific community, taken together with new immunohistochemical findings and specific recommendations for diagnostic pathology.

## Consent

Written informed consent was obtained from the patient for the publication of this report and any accompanying images.
